The article "Exploration on the Cultivation of Undergraduates' Entrepreneurship Ability from the Perspective of Mental Health Education" was published in 2022. Journal: J Healthc Eng.

# Exploration on the Cultivation of Undergraduates' Entrepreneurship Ability from the Perspective of Mental Health Education

**DOI:** 10.1155/2022/9668220

**Published:** 2022-03-16

**Authors:** Jian Cao

**Affiliations:** ^1^Culture and Social Development College, Chongqing 400700, China; ^2^Chongqing Electric Power College, Chongqing 400053, China

## Abstract

Entrepreneurship is a test of people's knowledge and specific application ability, especially the psychological quality of entrepreneurs. In the process of starting a business, people's psychological qualities have a very important influence on the ultimate success of starting a business. The significance of cultivating college students' entrepreneurial psychological quality lies in that it is not only the requirement of the development of the times but also the realistic requirement of improving college students' entrepreneurial ability. Therefore, it is of great practical significance to bring the cultivation of college students' entrepreneurial psychological quality into entrepreneurship education. Good entrepreneurial psychological quality is the cornerstone of the building of entrepreneurship, which can lay the foundation for entrepreneurship and support the whole entrepreneurial process. Because of the importance of entrepreneurial psychological quality in the process of entrepreneurship, it is necessary to analyze the entrepreneurial psychological quality of college students and guide and cultivate them correctly. Based on this, this paper analyzes the penetration of mental health education in the cultivation of College Students' entrepreneurship education, which has a strong practical significance.

## 1. Introduction

As the main force of social entrepreneurship, it is particularly important for college students to carry out entrepreneurship education, and the key factor affecting the success of college students' entrepreneurship is good entrepreneurial psychological quality [1]. Entrepreneurship is a process in which human beings use knowledge and the ability to create a career through thinking innovation. Entrepreneurship is a comprehensive test of people's quality, especially the test of people's psychological quality [2]. Entrepreneurship is a test of people's knowledge and their specific application ability, especially a test of the psychological quality of entrepreneurs [3]. Entrepreneurial psychological quality refers to the physical and mental organizational elements, structure, and quality level formed and developed under the influence of environment and education, which are fully and steadily displayed and play a role in entrepreneurial social practice [4]. In the process of starting a business, people's psychological qualities have a very important influence on the success of starting a business [5]. Under the new format of “mass entrepreneurship,” college students, as an important part of the entrepreneurial team, have a subtle influence on the overall planning of enterprise development, restricting the future development of enterprises and determining the ultimate success or failure of entrepreneurship [6]. Compared with foreign college students' entrepreneurship development, domestic college students' entrepreneurship has just started, so it is necessary to break through the shackles of ideas and traditional culture, strengthen the counseling of college students' entrepreneurial psychological quality, and continuously promote the cultivation of good entrepreneurial personality of college graduates [7]. It is helpful to alleviate the employment pressure of college students. The entrepreneurial ability of universities is conducive to solving the problem of difficult employment of college students. Entrepreneurial ability is a person's ability of self-survival and self-development in entrepreneurial practice. It is conducive to the realization of College Students' self-worth. Through independent entrepreneurship, college graduates can closely combine their interests with their careers and do what they are most interested in, willing to do, and think is most worth doing. It is conducive to the improvement of College Students' own quality. Good entrepreneurial psychological quality, like the cornerstone of an entrepreneurial building, can lay the foundation of a career and support entrepreneurial life. Therefore, cultivating college students' good entrepreneurial psychological quality is the premise and key of entrepreneurship education.

The article "Exploration on the Cultivation of Undergraduates' Entrepreneurship Ability from the Perspective of Mental Health Education" was published in 2022. Journal: J Healthc Eng.

College students' entrepreneurial process is the process of creating a career by using their professional skills and abilities learned in college and then innovating their thinking [8]. Entrepreneurship is a test of college students' overall quality, especially a test of their psychological quality. Good entrepreneurial psychological quality is the cornerstone of this building, which can lay the foundation of entrepreneurship and support the whole entrepreneurial process [9]. College students' entrepreneurial psychological quality is characterized by a lack of firmness in belief, a lack of patience and tenacity in passion, and a lack of experience and courage in innovation. College students should have psychological qualities such as independence and cooperation, courage and restraint, and tenacity and adaptability [10]. Nowadays, the problem of mental health education has gradually attracted the attention of the education sector, especially in today's increasingly fierce competition, and the requirements for the quality and specifications of talents have gradually improved [11]. Therefore, students should vigorously carry out innovation and entrepreneurship education, cultivate students' entrepreneurial awareness and entrepreneurial ability, and infiltrate mental health education to enhance students' learning ability and practical ability [12].

College students do need not only a feasible entrepreneurial plan, excellent team and financial support, but also good entrepreneurial psychological quality [13]. Therefore, it is of great practical significance to bring the cultivation of college students' entrepreneurial psychological quality into entrepreneurship education. The significance of cultivating college students' entrepreneurial psychological quality is that it is not only the requirement of the development of the times but also the realistic requirement of improving college students' entrepreneurial ability [14]. Entrepreneurial psychological quality exerts a subtle influence on the development and survival of new ventures and also has a certain restrictive effect on the comprehensive competitiveness of enterprises [15]. Cultivating college students' entrepreneurial psychological quality has important theoretical and practical significance for promoting the all-round development of college students, promoting the effective development of college students' entrepreneurial activities and improving the success rate of college students' entrepreneurship [16]. The mature psychological quality of entrepreneurship is the cornerstone of entrepreneurial activities, which can lay the foundation for entrepreneurship and play an important supporting role in the process of entrepreneurship [17]. It is precise because of the importance of entrepreneurial psychological quality in the process of starting a business that it is necessary to analyze the entrepreneurial psychological quality of college students when starting a business and guide and cultivate it correctly [18]. Based on this, this paper analyzes the infiltration of mental health education in the cultivation of college students' entrepreneurship education, which has strong practical significance.

This paper analyzes the penetration of mental health education in college students' entrepreneurship education, which has strong practical significance. The innovative contributions of this paper are as follows: (1) The infiltration of mental health education into entrepreneurship education can not only realize the innovation of teaching mode and enrich teaching content but also enhance the effectiveness of education. (2) Mental health education can assist entrepreneurship education and enable students to participate in entrepreneurial activities under the condition of mental health. The improvement of College Students' entrepreneurial psychological quality should be the result of the joint efforts of all parties. (3) Colleges and universities should deal with the relationship between College Students' mental health education and the improvement of College Students' entrepreneurial ability, explore the best combination of the two, and explore new ways to improve college students' entrepreneurial ability through college students' mental health education.

The article "Exploration on the Cultivation of Undergraduates' Entrepreneurship Ability from the Perspective of Mental Health Education" was published in 2022. Journal: J Healthc Eng.

This paper is divided into four parts. The first part expounds the background of mental health education in college students' entrepreneurship education. The second part studies the significance of mental health education in the cultivation of College Students' entrepreneurship education. It has stimulated college students' entrepreneurial enthusiasm and improved college students' psychological quality. The third part expounds the training path of College Students' entrepreneurial ability from the perspective of mental health education. It improves college students' entrepreneurial cognitive ability and cultivates college students' entrepreneurial group cooperation consciousness.

## 2. The Significance of Psychological Health Education in the Cultivation of College Students' Entrepreneurship Education

### 2.1. Stimulating the Entrepreneurial Enthusiasm of College Students

With the development of China's social economy, college education has gradually changed from elite education to mass education, and the employment positions that society can provide for college students are relatively reduced. This requires college students to dare to face challenges and start their own businesses. With the development of information technology and network technology in China, various educational activities are constantly innovating in form and concept to a certain extent. Combining with the development trend of the times, infiltrating mental health education into innovative education can not only realize the innovation of teaching mode and enrich teaching content, but also improve the effect of education and interpret the value of entrepreneurship education [19]. Through the practice of mental health education and group psychological counseling, students' learning motivation can be stimulated, and every college student's potential can be fully developed. Group psychological counseling in mental health education meets this need and will continue to play an important role in cultivating college students' collective cooperation consciousness and win-win team concept. In the field of psychological education, its main content is mental health knowledge, which has many details. When students' mental health knowledge structure is improved, their psychological quality can be improved.

The article "Exploration on the Cultivation of Undergraduates' Entrepreneurship Ability from the Perspective of Mental Health Education" was published in 2022. Journal: J Healthc Eng.

In entrepreneurial activities, the scale of social relations, which is an important factor of social capital, has the most important influence on entrepreneurial performance. Entrepreneurs with a large scale of social relations have strong financing ability and can decide their own investment behavior independently according to market opportunities, thus improving the success rate of entrepreneurship. The specific process can be shown in Figure 1. Firstly, the minimum spanning tree is obtained, and then the loop is controlled according to the condition, and the edge with the largest weight is cut off. If you need to get two clusters, you only need to cut off one of the longest edges.

To a great extent, college students' entrepreneurship is a contest of psychological quality. Good entrepreneurial psychological quality is the subjective premise that affects whether college students can successfully transform from potential entrepreneurs to real entrepreneurs, and it is also the key that restricts the success of college students' entrepreneurship. For example, Table 1 shows the empirical analysis results of social entrepreneurship policy and entrepreneurial attitude.

The risk index system of the innovation and entrepreneurship team is established, and the risk is evaluated by AHP. The judgment matrix of weights is constructed. The data relationship between weight value and evaluation value is shown in the figure.  Figure 2 shows the data relationship between financial risk weight value and evaluation value.

In the new era, it is particularly important for college entrepreneurs to have team spirit and team cooperation consciousness. However, college students who are engaged in innovation and entrepreneurship now have strong self-awareness, and it is difficult to recognize the important role of college students' cooperative awareness in college students' entrepreneurship. Exercising and cultivating self-awareness of teamwork, expanding and developing self-network resources, which is not only a major issue to be solved urgently in school mental health education, but also one of the important contents that can not be ignored in contemporary college students' entrepreneurship education [20]. In order to cultivate innovative talents, it is necessary to strengthen the guidance of entrepreneurial psychological quality, improve the personality education of college students and improve their psychology so as to improve their entrepreneurial ability and make their employment ideas change from equal and dependent to active employment [21]. If they do not have good psychological quality, their entrepreneurial behavior will increase many barriers. From this point of view, the reasonable degree of mental health education will also have an impact on the effect of entrepreneurship education, and at the same time, it can also reflect the penetrating significance of mental health education in the cultivation of entrepreneurship education for college students.

The article "Exploration on the Cultivation of Undergraduates' Entrepreneurship Ability from the Perspective of Mental Health Education" was published in 2022. Journal: J Healthc Eng.

### 2.2. Improving the Psychological Quality of College Students

Psychological quality is both the foundation and the core. Psychological quality determines a person's performance and behavior, which is the same for college students. College students' mental health education is conducive to college students' understanding of their mental health level, a better understanding of themselves, self-understanding, and accurate self-positioning. Entrepreneurial psychological quality is the subjective premise factor that affects people's entrepreneurship, and it is also the key factor and important guarantee that restricts people's entrepreneurial success. Therefore, the cultivation of entrepreneurial psychological quality will become the core and key of entrepreneurship education. For college students, they need to go deep into society after graduation, and their status has changed from students to social citizens. This change in environment and identity will also lead to some ideas in their hearts. Some schools have carried out entrepreneurship education and training, but students cannot really devote themselves to entrepreneurial activities after learning [22]. The process of starting a business is not smooth sailing. Colleges and universities should enrich various second-class activities and focus on cultivating students' determination and perseverance in the face of difficulties and their positivity and optimism in the depths and valleys to enhance their ability to resist setbacks. The actual market situation is far more complicated than the competition situation in schools, and customers are not judges of schools. The judges will consider students' enthusiasm and self-confidence when making comments and point out problems politely. However, when customers are dissatisfied with products, they will directly choose other products. Innovation and entrepreneurship, as a high-risk entrepreneurial practice for college students, cannot bear the strong frustration caused by college students' entrepreneurial failure without certain psychological endurance.

After thousands of years of history, the Confucian culture has gradually become a collection of orthodoxy, shaping the overall social character, mode of thinking, norms, and psychological environment of the Chinese people. The content of Confucian culture is profound. As an ethical and moral system to maintain the traditional social order and moral people, the wisdom and value orientation contained in the essence of Confucian culture still have great guiding significance for today's society. Being good at excavating the coincidence point between mental health education and Confucian culture has important theoretical and practical value for enhancing mental health education, which is conducive to correctly understand and solve a series of practical problems of mental health education.

The article "Exploration on the Cultivation of Undergraduates' Entrepreneurship Ability from the Perspective of Mental Health Education" was published in 2022. Journal: J Healthc Eng.

Confucianism not only does not shy away from talking about emotion but also puts emotion in an important position in its theory. The Confucian psychological model regards the unity of beauty and goodness as the highest realm of life and advocates the high unity of art and ethics.  Figure 3 is an overview model of the Confucian psychological model.

For psychological evaluation, whether to achieve the purpose of psychological evaluation is an important basis for measuring the success or failure of work. The energy of the state can be defined as follows:

(1) $$\begin{array}{c} w_{ij}=w_{ij}+a\left(\frac{X_{i}}{m}-w_{ij}\right). \end{array}$$

Use bee colony optimization algorithm to mine data in depth, and use secondary correction function:

(2) $$\begin{array}{c} o_{k}=f\left({\text{net}}_{k}\right),\\ {\text{net}}_{k}=\sum_{j=0}^{m}w_{jk}y_{j},\\ y_{j}=f\left({\text{net}}_{j}\right),\\ {\text{net}}_{j}=\sum_{i=0}^{n}v_{ij}y_{j}. \end{array}$$

By being a polynomial kernel function:

(3) $$\begin{array}{c} E_{\text{RME}}=\sqrt{\frac{1}{P}\sum_{p=1}^{P}{\left(E_{P}\right)}^{2}}. \end{array}$$

When the parameters are fixed, simplify it to the following:

(4) $$\begin{array}{c} \delta_{k}^{o}=\left(d_{k}-o_{k}\right)\left(1-o_{k}\right)o_{k},\\ \delta_{j}^{y}=\left[\sum_{k=1}^{l}\left(d_{k}-o_{k}\right)f\prime \left({\text{net}}_{k}\right)w_{jk}\right]f\prime \left({\text{net}}_{j}\right)\\ =\left(\sum_{k=1}^{l}\delta_{k}^{o}w_{jk}\right)\left(1-y_{j}\right)y_{j}. \end{array}$$

Construct a high-dimensional feature distribution space to represent the parameter index distribution model of psychological evaluation:

(5) $$\begin{array}{c} \Delta w_{jk}=\eta \delta_{k}^{o}y_{j}\\ =\eta \left(d_{k}-o_{k}\right)\left(1-o_{k}\right)o_{k}y_{j},\\ \Delta v_{ij}=\eta \delta_{j}^{y}x_{i}\\ =\left(\sum_{k=1}^{l}\delta_{k}^{o}w_{jk}\right)\left(1-y_{j}\right)y_{j}x_{i}. \end{array}$$

If we want to establish the norm of the Confucian psychological model, we must take theory as the guiding principle. This theoretical principle should be cognitive schema theory because it is a theory that reveals people's cognitive characteristics. Taking the statistical results of the psychological model parameters of Confucianism as the research object, we deal with data clustering and information fusion.  Table 2 shows the test results of the indicators.

The article "Exploration on the Cultivation of Undergraduates' Entrepreneurship Ability from the Perspective of Mental Health Education" was published in 2022. Journal: J Healthc Eng.

In order to better study the influence of price competition on various factors, the demonstration part adopts the idea of the normalization of price competition degree. The evaluation indexes of talent training are divided. The specific division is shown in Table 3.

Due to the inadequate construction of various links in asset management of state-owned enterprises, an effective communication and liaison mechanism has been established among internal departments of state-owned enterprises. Calculate the geometric mean of all elements in each row in the judgment matrix:

(6) $$\begin{array}{c} n=\sum_{i-1}^{R}P_{l}W_{l,j}+b. \end{array}$$

Get the following:

(7) $$\begin{array}{c} E_{p}=\frac{{\sum \left(t_{pi}-o_{pi}\right)}^{2}}{2}. \end{array}$$

Calculate the random consistency ratio:

(8) $$\begin{array}{c} E_{p}=\frac{{\sum \left(t_{pi}-o_{pi}\right)}^{2}}{2}. \end{array}$$

Contemporary entrepreneurial college students generally lack practical experience, and their knowledge comes from books, lectures, etc., rather than reality, which is often a fatal problem after joining the career. Schools should attach great importance to the education of mental health knowledge and provide timely and effective psychological counseling to students. Once it is found that external factors have affected their emotions, they should reasonably channel students' moods to avoid the influence of bad psychology on students' life and work. As an important part of quality education, mental health education should run through the whole process of higher education [23]. This is the realistic need to promote college students' personality psychology, entrepreneurial will, develop and cultivate sound personality, and it is also the need to face and adapt to future economic and social market competition. Edison tried more than 3,000 different filament materials but failed. But he was never discouraged, and it was this indomitable spirit that helped him succeed. If college students want to start their own businesses, they must also have this kind of resilience and be able to maintain a high-spirited and enterprising attitude after repeated failures. To simulate the entrepreneurial process, we should pay attention to psychological changes, clarify students' ideas, and give dynamic observation to improve their ability, improve their entrepreneurial structure, give full play to their subjective initiative, and realize the hardships of entrepreneurship.

The article "Exploration on the Cultivation of Undergraduates' Entrepreneurship Ability from the Perspective of Mental Health Education" was published in 2022. Journal: J Healthc Eng.

## 3. The Path of Cultivating College Students' Entrepreneurial Ability from the Perspective of Mental Health Education

### 3.1. Improving College Students' Entrepreneurial Cognitive Ability

At present, the frequency and quantity of psychological problems among college students are obviously on the rise, so the relevant departments and leaders of the school should find out the students' problems as early as possible, prevent them as early as possible, and try their best to reduce the probability of mental health problems. In order to achieve a good “match” between college students' individual and entrepreneurial choices, they must accurately position themselves on the basis of fully understanding their entrepreneurial ability. After students enter school, schools should investigate students' psychology. Besides, they can also use the opportunity of face-to-face communication between students and counselors to fully grasp students' psychological conditions and use professional psychotherapy methods to help students solve psychological obstacles and eliminate bad emotions. Scientific professional psychological counseling plays a certain role in cognitive adjustment and value guidance in the process of college students' entrepreneurship. It can enable college entrepreneurs to set up scientific career planning, clarify the development direction of self-entrepreneurship, and learn to use scientific career planning knowledge to solve many psychological puzzles that may be encountered in the process of entrepreneurship so as to optimize psychological quality and achieve entrepreneurial goals. From reality, in the process of starting a business, personality is very important and crucial, and most successful entrepreneurs have unique personality charm, which shows the importance of personality [24]. We should actively explore the entrepreneurial resources of outstanding entrepreneurs, especially outstanding alumni, and invite them to come to the school to give their own opinions to college students so that college students can choose their social needs, their own love and their own strengths in entrepreneurial practice. At the same time, it will also strengthen college students' entrepreneurial ideals and establish their confidence in the success of entrepreneurship. In the process of mental health education, teachers should guide students' behavior and psychology correctly so that they can actively participate in team activities, exercise their ability to adapt to society, and constantly form a strong will to participate in various activities reasonably. In the long run, students can learn to restrain their bad behaviors, control their bad emotions, and deal with various problems with a very positive attitude.

The article "Exploration on the Cultivation of Undergraduates' Entrepreneurship Ability from the Perspective of Mental Health Education" was published in 2022. Journal: J Healthc Eng.

According to the theory of planned behavior, the more positive the attitude and subjective norms are, the stronger the control of perceived behavior is, and the stronger the individual's intention to consider executing behavior is. The data relationship between weight value and evaluation value is shown in Figure 4.

Taking the statistical results of big data, an index parameter of psychological evaluation, as the research object, data clustering, and information fusion are carried out to realize the evaluation of evaluation ability. A comparison of the two analysis methods is shown in Figure 5.

In order to start a business, college students can have good psychological quality when starting a business, and they can start to educate students' entrepreneurial psychology during their college years. Colleges and universities should integrate entrepreneurial psychology education into teaching, set up a professional team of teachers of entrepreneurial psychology education, so as to intervene in time the psychological problems of students when starting a business, and provide professional entrepreneurial consultation and help. College students must have a positive attitude in starting a business so that they can spread their enthusiasm to others and make a good impression on customers. If we want to cultivate students' positive mentality, we should give the appropriate guidance and encourage students to find the reasons for failure as soon as possible after problems arise, instead of evading responsibility [25]. Carrying out entrepreneurial practice gradually shows its advantages in cultivating entrepreneurial college students' psychological quality. Students can not only train their professional skills and cultivate core technologies in entrepreneurial practice but also cultivate their psychological quality, anti-stress ability, innovative spirit and courage. For psychological counselors, they should give targeted guidance to students according to their specific characteristics and provide consulting services for students. Especially for some students with psychological problems, they should conduct an in-depth investigation of their data, establish personal files, and make clear the causes of students' psychological problems in time. Colleges and universities should focus on cultivating students' independent consciousness and ability to solve problems alone. In the daily study, life, and second class activities, teachers only play the role of instructors, encouraging students to find answers and solve problems independently, and providing students with enough room for growth and development.

The article "Exploration on the Cultivation of Undergraduates' Entrepreneurship Ability from the Perspective of Mental Health Education" was published in 2022. Journal: J Healthc Eng.

### 3.2. Cultivating College Students' Awareness of Cooperation in Entrepreneurial Groups

For some students with strong entrepreneurial motivation, entrepreneurship psychological education should be targeted to improve students' psychological quality and deal with the problems in the process of entrepreneurship. Group psychological counseling is a form of mental health education conducted under the group situation. Through interpersonal interaction within the group, it promotes individual college students to adjust and improve their relationship with others by observing, learning, experiencing, knowing, exploring, and accepting themselves. The formation of good entrepreneurial psychological quality focuses on practical training. Active practice can bring timely feedback and a sense of accomplishment and also bring the joy of continuous success so that college students can put themselves into entrepreneurial practice and hone their strong entrepreneurial psychological quality. Entrepreneurship is not the choice of all college students, but there are still some students in college students who are suitable for entrepreneurship. For these students, they need to provide entrepreneurial help. Students will put forward psychological needs in the process of entrepreneurship, and at the same time, they will have some psychological problems [26]. Generally speaking, the degree of monopoly in the market structure is positively correlated with the scale of enterprises. This means that the higher the degree of monopoly in the market structure, the larger the scale of enterprises, the stronger the ability of enterprises to carry out technological innovation, and vice versa. Economic monopoly, enterprise-scale, and technological innovation capability are shown in Figure 6.

In college students' group psychological counseling activities, we can set up a variety of activity programs, let more people participate in the discussion and divide them into several groups to contract and cooperate, participate in and complete a large-scale activity together, and give full play to the subjective initiative of each entrepreneurial member. Only through the practice of entrepreneurship can the goal of entrepreneurship become clearer, the belief of entrepreneurship become stronger, and then form good entrepreneurial habits and personality.  Figure 7 shows the network structure system of talent entrepreneurship awareness management.

Teachers can play a leading role in the training system of college students' entrepreneurship education, so teachers must pay attention to the related problems of students' psychological regulation so as to improve the mental health education system. Colleges and universities should plan, design, and organize entrepreneurial practice activities, combine extracurricular activities and collective individual activities, and strengthen the entrepreneurship awareness education of college students, so that those students with active thinking, well-informed information, and strong practical operation ability can carry out entrepreneurial simulation practice as soon as possible so that they can successfully enter the ranks of college students' entrepreneurship after graduation. Teachers need to pay attention to students' psychological control ability in the process of entrepreneurship education and summarize the existing problems in time to help students face difficulties and setbacks with a positive attitude in the fierce social competition. If some students' self-confidence in innovation and entrepreneurship cannot be improved, it is necessary to further improve the mental health education system in combination with the current actual situation.

The article "Exploration on the Cultivation of Undergraduates' Entrepreneurship Ability from the Perspective of Mental Health Education" was published in 2022. Journal: J Healthc Eng.

## 4. Conclusions

Good entrepreneurial psychological quality is the cornerstone of college students' successful entrepreneurship, which can lay the foundation for their careers and support their entrepreneurial life. Infiltrating mental health education into entrepreneurship education can not only realize the innovation of teaching mode and enrich teaching content, but also enhance the substantive effect of education. Psychological health education can assist entrepreneurship education so that students can participate in entrepreneurship activities under the condition of mental health. The promotion of college students' entrepreneurial psychological quality should be the result of joint efforts of all parties. It needs the influence of social environment, professional education in colleges and universities, family care and support, and the promotion of college students' self-awareness. Colleges and universities should deal with the relationship between mental health education of college students and the promotion of entrepreneurial ability of college students, explore the best fit between them, and explore a new way to promote the entrepreneurial ability of college students by exerting mental health education of college students. College students should establish a correct understanding, maintain a healthy mentality, and gradually improve their entrepreneurial psychological quality with the help and support of society, schools, and families so as to lay a good foundation for participating in innovation and entrepreneurship and realizing their entrepreneurial dreams. [27].

The article "Exploration on the Cultivation of Undergraduates' Entrepreneurship Ability from the Perspective of Mental Health Education" was published in 2022. Journal: J Healthc Eng.

## Figures and Tables

**Figure 1:** Spanning tree process.

**Figure 2:** Data relationship between weight value and evaluation value.

**Figure 3:** Overview model.

**Figure 4:** Data relationship between weight value and evaluation value.

**Figure 5:** Comparison of accuracy data of two analysis methods.

**Figure 6:** The relationship between economic monopoly, enterprise-scale, and technological innovation capability.

**Figure 7:** Network structure system of talent entrepreneurship awareness management.

**Table 1:** Empirical analysis results of social entrepreneurship policy and entrepreneurial attitude.

Variable	Perceptual skills	Perceived opportunity	Entrepreneurial intention	Fear of failure
Entrepreneurial support	0.077	0.155	0.069	0.264
Entrepreneurship education	0.059	0.248	0.054	0.381
Entrepreneurial environment	0.012	0.081	0.038	0.042
Type of economy	0.017	0.082	0.096	0.041

**Table 2:** Evaluation test data.

Stage	1	2	3	4	5	6
Frequency	80.31	88.52	74.77	88.52	81.97	72.84
Accuracy	70.59	78.78	85.64	87.96	76.35	88.29

**Table 3:** Classification of talent training evaluation.

Personnel training evaluation parameters	0–20	20–25	25–30	35–40	40–45
Normalized value	0.2	0.25	0.3	0.4	0.45

## Data Availability

The data used to support the findings of this study are included within the article.
